# Phyto-Extract-Mediated Synthesis of Silver Nanoparticles (AgNPs) and Their Biological Activities

**DOI:** 10.1155/2022/9845022

**Published:** 2022-11-16

**Authors:** Muhammad Adnan, Asma Akbar, Sakina Mussarat, Waheed Murad, Ishfaq Hameed, Shaheen Begum, Ruqia Nazir, Nawab Ali, Essam A. Ali, Ahmed Bari, Muhammad Abdul Aziz, Shahid Niaz Khan

**Affiliations:** ^1^Department of Botany, Kohat University of Science and Technology, Kohat 26000, Pakistan; ^2^Department of Botany, Abdul Wali Khan University Mardan, Pakistan; ^3^Department of Botany, University of Chitral, Chitral 17200, Pakistan; ^4^Department of Environmental Sciences, Fatima Jinnah Women University, Rawalpindi, Pakistan; ^5^Department of Chemistry, Kohat University of Science and Technology, Kohat 26000, Pakistan; ^6^Department of Biotechnology and Genetic Engineering, Kohat University of Science and Technology, Kohat 26000, Pakistan; ^7^Department of Pharmaceutical Chemistry, College of Pharmacy, King Saud University, Riyadh 11451, Saudi Arabia; ^8^Department of Environmental Sciences, Information and Statistics, Ca Foscari University of Venice, Vio Tornio 155, 30172 Venezia, Italy; ^9^Department of Zoology, Kohat University of Science and Technology, Kohat 26000, Pakistan

## Abstract

**Background:**

Nanotechnology finds broad applications in the field of nanomedicine, an emerging new field used for diagnosis, treatment, prevention of diseases, and improvement of health.

**Objectives:**

To synthesize silver nanoparticles (AgNPs) from *Withania somnifera* and *Fagonia indica* and to carry out their antimicrobial, insecticidal, and phytotoxic activities, a step toward the new range of nanomedicines.

**Methods:**

Silver nanoparticles were synthesized from *Withania somnifera* and *Fagonia indica* by chemical reduction method, and further biological activities of these nanoparticles were compared with crude methanolic extract, prepared through cold maceration process, at the concentration of 50 mg/ml.

**Results:**

Among all tested bacterial pathogens, crude extract of *W. somnifera* showed a statistically high significant inhibition zone in millimeter against *Pseudomonas aeruginosa* (21; *p* < 0.01). AgNPs showed highly significant result against *Streptococcus pneumonia* (14; *p* < 0.01). In comparison with crude extracts, AgNPs showed statistically significant (*p* < 0.01) results against *S. pneumonia* (AgNPs, 14; crude, 8.33 mm). Crude extract showed significant inhibition zone against two bacterial strains, *P. aeruginosa* (crude, 21; AgNPs, 11.67 mm) and *Klebsiella pneumoniae* (crude, 11.33; AgNPs, 8 mm). Crude extracts of *F. indica* showed the significant activity against *Vibrio cholera* (*p* < 0.01; 11.33 mm). Silver nanoparticles of *F. indica* exhibited the highest significant activity against *Aspergillus flavus* and *Fusarium oxysporum* while AgNPs of *W. somnifera* were active only against *A. flavus*. Extracts of *W. somnifera* and *F. indica* showed increasing phytotoxic activity with increasing concentrations. The highest significant inhibition was obtained for crude extract (46.7) and AgNPs (45.7) of *F. indica* at 1000 *μ*g/ml. Insecticidal activity of crude and AgNPs of both plants showed significant inhibition against all tested insects with increasing time intervals, and the highest significant result was obtained at 72 hours with a value of *p* < 0.01 except *T. castaneum*.

**Conclusions:**

Both crude and AgNPs showed potent activity; however, in comparison, silver nanoparticles showed slightly enhanced activity. Crude and AgNPs of both plants showed good phytotoxic and insecticidal inhibition. Antimicrobial studies of AgNPs on diseases causing pathogens open a door for new antimicrobial agents and could be the answer to antibiotic resistance after further analysis.

## 1. Introduction

Plants used as medicines to treat different diseases are a rich source of various bioactive components like volatile tannins, oils, alkaloids, flavonoids, and phenols which have a prominent role in the discovery of new drugs to treat infectious diseases. Many scientists have isolated and characterized different pharmacologically dynamic compounds from traditionally used medicinal plants. With the progress of drug development, there is a need to utilize advanced technology such as nanotechnology which has tremendous application in the pharmaceutical industries [1]. Nanotechnology finds broad applications in the field of nanomedicine, an emerging new field used for diagnosis, treatment, prevention of diseases, and improvement of health. Due to specific characteristics of nanoparticles such as small size, distribution, and morphology, these have new applications and properties. Nanoparticles can be synthesized by different methods like chemical and photochemical reactions [2], thermal decomposition [3], and microwave assisted process [4] and also by biological methods [5, 6]. Both in the medical and industrial processes, silver has a good inhibitory effect on microbes, and silver nanoparticles have applications in the medical industry such as in topical ointments to prevent infection of burn and wounds as well as prevent bacterial contamination in humans [7]. Nowadays, silver nanoparticles (AgNPs) have interesting antibacterial activities and have played a crucial role in inhibiting bacterial growth in aqueous and solid media [8, 9] and may be an answer to bacterial resistance, caused by the overuse of antibiotics. *Withania somnifera* (L.) Dunal (Solanaceae), a commonly used plant in traditional and Ayurvedic medicine, has withanolide-type active compounds and is widely used in crude form throughout the world due to its nontoxic and high medicinal value. Nowadays, this plant is cultivated as a crop to support the high demand for biomass and fulfill the needs of pharmaceutical industry. Similarly, *Fagonia indica* Burm.f. (*Zygophyllum indicum* (Burm.f.) Christenh. & Byng) is a small spiny herb widely used in Ayurvedic medicine belonging to Zygophyllaceae having analgesic, antimicrobial, febrifuge, and anti-inflammatory properties with active phytoconstituents [10]. The present study has been designed to synthesize AgNPs by using *W. somnifera* and *F. indica* extract and to carry out the antimicrobial, insecticidal, and phytotoxic activities and their comparison with the crude extract, a step toward the new range of antimicrobial agents in the field of nanomedicine.

## 2. Materials and Methods

### 2.1. Collection and Formulation of Plant Extracts

*F. indica* and *W. somnifera* were collected from Karak and Kohat, identified by the taxonomist at the Department of Botany, Kohat University of Science and Technology, Kohat. Collected plant parts were washed, dried in shade, powdered, and stored in airtight bottles. The crude methanolic extract was prepared through cold maceration extraction technique and further used for biological activities.

### 2.2. Synthesis of Silver Nanoparticles (AgNPs)

Chemical reduction method was used to synthesize the silver nanoparticles (AgNPs) of *F. indica* and *W. somnifera* [11]. 1 ml of silver nitrate solution was diluted; then, 100 g of both plant extracts was dissolved in 100 ml of deionized water. Both the plant extracts and silver nitrate solution were mixed in 1 : 1 in a beaker. A homogeneous solution was obtained when this mixture was stirred and placed on a hot plate. After that, a reducing agent Sodium Borohydrate (NaBH_4_) was added dropwise through a burette with a constant stirring. The formation of silver nanoparticles was finished when the solution color was changed from light brown to dark.

### 2.3. Antibacterial Assay

Eight bacterial strains *Escherichia coli*, *Salmonella typhimurium*, *Shigella flexneri*, *Proteus mirabilis*, *Streptococcus pneumonia*, *Pseudomonas aeruginosa*, *Vibrio cholera*, and *Klebsiella pneumonia* and all the ATCC cultures except *S. flexneri* and *V. cholera* that were hospital-acquired clinical isolates were obtained from the laboratory of Department of Microbiology, and antibacterial activities were determined by Agar Well diffusion method [12] at 50 mg/ml concentration. Dimethyl sulfoxide (DMSO) was used as negative control while ampicillin as a positive control. Experiments were repeated three times, and average zones of inhibition were recorded.

### 2.4. Antifungal Assay

Two fungal strains *Aspergillus flavus* and *Fusarium oxysporum* were obtained from the laboratory of Department of Microbiology. Test tube dilution method, with slight modification, was followed to check the antifungal activities [13], and 6.5 g of Sabouraud Dextrose Agar (SDA) was mixed in 100 ml of distilled water and autoclaved, and 9 ml of this mixture was taken in a test tube. Every test tube was loaded with 1 ml of extract solutions before solidifying. The tubes were inoculated with a 4 mm diameter piece of the fungal pathogen, allowed to solidify, and placed in a slanting position in an incubator at 28°C for 7 days. Miconazole was used as a positive control to compare the antifungal activity. The inhibition zone was measured in millimeter.

### 2.5. Phytotoxic Activity

Phytotoxic activity was carried out against *Lemna minor* [14]. E-medium was prepared and autoclaved at 15 psi, 121°C for 15 minutes. Each plant extract of 30 mg (crude and silver nanoparticles) was then dissolved in methanol (1.0 ml) which served as a stock solution. Seven petri dishes were autoclaved, and 20 ml medium on each plate and 60 ml of plant extract having one frond of *Lemna minor* were added. Paraquat was used as a negative control, and plates were placed in a growth cabinet; the number of fronds per plate was counted and recorded, and the experiment was repeated three times.

### 2.6. Insecticidal Activity

*Rhyzopertha dominica*, *Sitophilus oryzae*, *Callosobruchus analis*, and *Tribolium castaneum* were selected for the present study. Filter papers of 9 cm or 90 mm were cut out and put out on the plate. Plant extract (50 mg/ml) was poured over the filter papers, and then, these plates were left for almost one day. 10 healthy insects of equal size/age were put out on the second day of each species in each plate and were incubated at 27°C. Permethrin was used as a positive control. The results were noted after 24 hours, 48 hours, and 72 hours, respectively. Experiments were repeated three times.

### 2.7. Statistical Analysis

Data were organized and analyzed using Microsoft Word and Microsoft Excel software. All the experiments were repeated, and the average zone of inhibition and standard deviations were calculated by using Microsoft Excel software 2007. Significant values of all activities were found by using one-way ANOVA and *t-test*.

## 3. Results

### 3.1. Antibacterial Effect of Crude Extracts and Silver Nanoparticles

Among all tested bacterial pathogens, crude extract of *W. somnifera* showed highly significant inhibition against *P. aeruginosa* (21; *p* < 0.01), followed by *S. flexneri* (12.33 mm) and *K. pneumoniae* (11.33 mm). The lowest inhibitory activity was measured for the *S. typhimurium* (5 mm). The tested antibiotic is sensitive to this bacterium (25 mm). AgNPs also showed highly significant results against *S. pneumonia* (14; *p* < 0.01), followed by *P. mirabilis* (11.67 mm) and *P. aeruginosa* (11.67 mm) (Table 1). The lowest inhibition zone was measured for *S. typhimurium* (6.33 mm) as compared to the antibiotic inhibitory zone (25 mm). In the comparison of both extracts, AgNPs showed statistically highly significant (*p* < 0.01) results against *S. pneumonia* (AgNPs, 14; crude, 8.33 mm). Crude extract showed significant inhibition against two bacterial strains, *P. aeruginosa* (crude, 21; AgNPs, 11.67 mm) and *K. pneumonia* (crude, 11.33; AgNPs, 8 mm) (Table 1).

Crude extracts of *F. indica* showed the highest significant inhibition zone at *p* < 0.01 for *Vibrio cholera* (11.33 mm) followed by *S. pneumonia* (10.33 mm). The lowest inhibition zone was measured for the *E. coli* (7.00 mm). Similarly, AgNPs showed an inhibition zone ranging from 8.00 to 11.67 mm. The highest significant inhibition zone at *p* < 0.01 was measured for *S. flexneri* (11.67 mm) and *V. cholera* (11.67 mm) followed by *P. aeruginosa* (10.33 mm) and *E. coli* (10 mm) as compared to the antibiotic activity of 26 mm, 21 mm, 20 mm, and 22 mm, respectively.

### 3.2. Antifungal Activity of Crude Extracts and Silver Nanoparticles

AgNPs of *W. somnifera* exhibited the highest significant antifungal activity as compared to crude extract against *A. flavus* (12; *p* < 0.01). AgNPs of *F. indica* also showed statistically significant inhibition as compared to crude extract against both tested fungal strains (Table 2).

### 3.3. Phytotoxic Activity of Crude Extracts and Silver Nanoparticles

Phytotoxic activity of both plants showed increasing inhibition with the increasing concentration against the growth of the *Lemna minor*. Both extracts of *W. somnifera* crude and silver nanoparticles displayed the most important spectrum of activity, at the highest concentration 1000 *μ*g/ml, and silver nanoparticles, which is a nonsignificant value.

Statistically, all the treatments of *F. indica* are highly significant at the highest concentration of 1000 *μ*g/ml among crude and silver nanoparticles, individually (Table 3). The highest significant inhibition value (46.7) has been obtained on 1000 *μ*g/ml for the crude extract of *F. indica*. The highest significant value (45.7) has been obtained on treatment supplemented by silver nanoparticles at 1000 *μ*g/ml concentration. Overall, crude extract showed slightly enhanced activity but the comparison was nonsignificant.

### 3.4. Insecticidal Activity of Crude Extracts and Silver Nanoparticles

Crude extracts and AgNPs of *W. somnifera* were evaluated against the insects including *R. dominica*, *S. oryzae*, *C. analis*, and *T. castaneum* with different time intervals (24, 48, and 72 hours); significant differences were observed for both crude and AgNP treatment. Crude extract of *W. somnifera* showed significant inhibition against all tested insects with increasing time intervals while AgNPs showed significant inhibition against *S. oryzae* and *C. analis* (Figure 1). Crude extract and AgNPs of *F. indica* showed the highest significant value at 72 hrs (4.33 inhibition of insects) (*p* < 0.01) for all tested insects except *T. castaneum* (Figure 2).

## 4. Discussion

In the present study, both the crude and AgNP extracts of both selected plants, *W. somnifera* and *F. indica*, showed good inhibition against the bacterial, fungal, insecticidal, and phytotoxic activity. However, AgNPs showed slightly more inhibition against bacterial and fungal strains than crude extract. AgNPs synthesized from *W. somnifera* has a good antimicrobial effect against gram-positive, gram-negative, and fungal pathogens by breaking out the cell membrane of bacteria, as confirmed by SEM analysis [15]. These AgNPs are small, easily penetrate the cell, and target the disease site as well as damage the cellular structure of pathogenic microbes. AgNPs from the same family, Solanaceae, also showed effective antimicrobial activity against gram-negative bacteria [16]. A group of monomeric glycoproteins, namely, WSG (*Withania somnifera* glycoprotein), isolated from *W. somnifera* roots tuber exposed the antimicrobial activities against bacterial and fungal isolates, and it is reported that nanoparticles encased with phytoconstituents can be more effective [17]. A study conducted by Malesh and Satish [18] investigated that *W. somnifera* extracts of methanol depicted significant antimicrobial activities against a group of bacteria. DNA replication weakening and inactivation proteins are the mechanisms behind the antimicrobial activity of metallic nanoparticles [19].

Antimicrobial approach for the AgNPs is due to the discharge of silver ions (Ag-) in the cells and attached bioactive constituents [20]. Govindaraju et al. [21] reported antimicrobial activity of synthesized silver nanoparticles against *P. aeruginosa*, *S. aureus*, *A. flavus*, and *A. niger*. Mechanisms involved are changing in cell membrane permeability [22], generation of a group of free radicals that are responsible for the cell membrane damage [23], and indulgence of the single proton (H+) attractive force responsible for the damage of the cell membrane [24], but the exact procedure has not been fully explained. Moreover, the effect of silver nanoballs on different bacteria, i.e., *E. coli*, *S. typhimurium*, *P. aeruginosa*, and *B. subtilis*, by the formation of colony forming unit (cfu) and growth rate at a different concentration of 40 lg/ml showed significant retardation of bacterial growth [25]. Numerous fungal strains showing drug resistance like *F. solani*, *Candida albicans*, *A. flavus,* and *Candida glabrata* have been reported for resistance [26]. A study conducted by Malesh and Satish [18] investigated that *W. somnifera* crude extracts depicted significant antifungal activities against *Aspergillus flavus*, *Drechslera turcica,* and *Fusarium verticillioides*. Vivek et al. [27] have also reported the antifungal activities of AgNPs and mechanisms to suggest that depending on composition, the cell wall can act as a barrier preventing drugs from reaching the site of action. Interaction between AgNPs and the membrane structure of *A. flavus* and *F. oxysporum* cells was confirmed and found out significant changes to their cell membrane integrity, due to the “pits” on their surface site and also the formation of pores, and causes death of a cell [28]. The positive charge on Ag+ may have potent toxicity or antimicrobial activities as it forms complexes with DNA/RNA and specifically interacts with the nucleosides [29]. Moreover, the electrostatic attraction among the negatively charged microbial cells and positively charged NP has been reported [30]. The Ag+ ions bind to the cytoplasm and cell wall due to electrostatic attractions and affinity for sulphur proteins, significantly increase the permeability, and cause disintegration of bacterial casing.

The field of allelopathy is a significant ecological factor in the kingdom Plantae together with such types of phytotoxic medicinal plants in which flavonoids and alkaloids are studied as allelochemicals [31]. *Lemna minor* inhibition variations by plants might be due to different types of plant extract, their different components, and mode of extraction [32]. Phytotoxic effects of nanoparticles on shrimp's larvae can be linked with anticancer activity, and nanoparticles could be an alternative source of anticancer drugs [33] Toxicological study of the crude extract regarding intracutaneous toxicity and acute systematic toxicity in experimental animal models shows toxic nature of plants. The toxicity of this plant and the mechanism of action cannot be explained until unequivocal identification of its constituents [34].

Insects are cosmopolitan and occupy more than two-thirds of the known species of the animal kingdom. Flora including medicinal plants is part of insect's food and also destroys them and other stored products causing a huge amount of loss to the food and food quality [35]. Nanotechnology is the modern approach for the better management of insects and pest control in agriculture. The larvicidal activity of *Azima* crude extract and AgNPs is 100% at 24- and 48-hour exposure periods which may be due to the interactions of the compounds [36]. Larvicidal activities of AgNPs using aqueous extract of *Eclipta prostrata* were studied against *Culex tritaeniorhynchus*, *Anopheles subpictus*, and *Diptera culicidae* and showed different inhibitions for a period of one day [37]. The extracts of *P. harmala* have an insect's mortality rate of 21.0%, followed by the medicinal plant of *F. cretica* 9.0% while *Tribulus terrestris* has 2.6%. All treatments from 5 to 20% showed validity in killing *T. castaneum*. Goswami et al. [38] reported the activity of different surface functionalized hydrophilic nanoparticles, against *S. oryzae*. Yang et al. [39] checked the activity of polyethylene glycol-coated nanoparticles loaded with garlic essential oil against adult *T. castaneum* and observed the control efficacy of about 80%, presumably due to the slow and persistent release of the active components from the nanoparticles. Khan et al. [40] reported the importance of nanoparticles and their mechanistic approach in the field of medicine to treat chronic diseases like cancer. Similarly, anticancer and antimicrobial activity of silver nanoparticles synthesized from *Conocarpus lancifolius* showed marked inhibition [41]. Gold nanoparticles from *Rauwolfia serpentina* showed antibacterial and antioxidant potential that have relevant results with the present study [42]. So, different types of nanoparticles can be used for efficient management in agriculture and formulation of new insecticides Although the standard drug used in comparison showed higher inhibition, the crude extracts of plants and AgNPs synthesized by chemical and biological methods are cost-effective and eco-friendly to use.

## 5. Conclusions

In conclusion, crude and AgNPs exhibit good effects; however, in comparison, AgNPs synthesized from both plants, i.e., *W. somnifera* and *F. indica*, showed enhanced inhibition against bacterial and fungal pathogens. In phytotoxic results, crude extracts of both tested plants are more effective as compared to AgNPs. Biological activities of AgNPs on tested pathogens open a door for new antimicrobial agents and could be the answer to antibiotic resistance as well nanomaterials in different forms can be used as an effective management in agriculture and formulation of new insecticides. The present study has provided a base for the researcher in the field of nanomedicine to synthesize and check the biological activities of nanoparticles and isolated compounds from other medicinal plants against other microorganisms. New antibiotics and therapeutics in nanoform should be made from these natural products and replaced with those showing resistance to microorganisms. Toxicology studies of these AgNPs should be recommended to ensure the safety. Studies on the comparison and characterization of silver nanoparticles to other phytochemicals need to be carried out.

## Figures and Tables

**Figure 1:** Insecticidal activity of crude and silver nanoparticles of *W. somnifera*. ^∗^ represents statistical significance (ANOVA); Ns: nonsignificant.

**Figure 2:** Insecticidal activities of crude and silver nanoparticles of *F. indica*. ^∗^ represents statistical significance (ANOVA); Ns: nonsignificant.

**Table 1:** Antibacterial zone of inhibition (mm) of crude and silver nanoparticles' extracts of *W. somnifera* and *F. indica* at 50 mg/ml concentration.

Bacteria	*W. somnifera*			*F. indica*			Control
	Crude (mean ± SD)	Silver nanoparticles (mean ± SD)	*T*-test	Crude (mean ± SD)	Silver nanoparticles (mean ± SD)	*T*-test	Antibiotic (AMP)
*E. coli*	10.67 ± 1.53	9.33 ± 1.15	Ns	7 ± 1	10 ± 1	Ns	22
*S. pneumonia*	8.33 ± 1.15	14 ± 1	*p* < 0.01	11 ± 1	9.67 ± 0.58	Ns	15
*S. flexneri*	12.33 ± 0.58	8 ± 1	*p* < 0.05	10 ± 1	11.67 ± 1.15	Ns	26
*P. mirabilis*	8.33 ± 0.58	11.67 ± 1.53	Ns	9.33 ± 0.58	8.67 ± 0.58	Ns	30
*P. aeruginosa*	21 ± 1	11.67 ± 1.15	*p* < 0.05	7.67 ± 0.58	10.33 ± 0.58	Ns	20
*V. cholera*	8 ± 1	9.33 ± 0.58	Ns	11.33 ± 1.53	11.67 ± 2.08	Ns	21
*K. pneumoniae*	11.33 ± 0.58	8 ± 1	*p* < 0.05	10 ± 1	8 ± 1	Ns	26
*S. typhimurium*	5 ± 1	6.33 ± 0.58	Ns	10.33 ± 1.53	9 ± 1	Ns	25
ANOVA	*p* < 0.01	*p* < 0.01		*p* < 0.01	*p* < 0.01		

Key: SD: standard deviation; AMP: ampicillin; Ns: nonsignificant.

**Table 2:** Antifungal zone of inhibition (mm) of crude and silver nanoparticles' extracts of *W. somnifera* and *F. indica* at 50 mg/ml concentration.

Fungus	*W. somnifera*			*F. indica*			Control
	Crude (mean ± SD)	Silver nanoparticles (mean ± SD)	*T*-test	Crude (mean ± SD)	Silver nanoparticles (mean ± SD)	*T*-test	Miconazole
*A. flavus*	7.67 ± 1.15	12 ± 1	*p* < 0.01	7.67 ± 0.58	13 ± 1	*p* < 0.05	22
*F. oxysporum*	11 ± 1	12.67 ± 0.58	Ns	8.33 ± 0.58	13 ± 1	*p* < 0.01	25

**Table 3:** Phytotoxic activity of crude and silver nanoparticles' extracts of *W. somnifera* and *F. indica* against *Lemna minor*.

*W. somnifera*								*F. indica*							
Crude (mean ± SD)			ANOVA	Silver nanoparticles (mean ± SD)			ANOVA	Crude (mean ± SD)			ANOVA	Silver nanoparticles (mean ± SD)			ANOVA
Concentrations				Concentrations				Concentrations				Concentrations			
10 *μ*g/ml	100 *μ*g/ml	1000 *μ*g/ml		10 *μ*g/ml	100 *μ*g/ml	1000 *μ*g/ml		10 *μ*g/ml	100 *μ*g/ml	1000 *μ*g/ml		10 *μ*g/ml	100 *μ*g/ml	1000 *μ*g/ml	
42.3 ± 2.5	45 ± 2	47.3 ± 2.5	Ns	42 ± 2	44 ± 1.7	45.3 ± 0.5	Ns	41.3 ± 1.1	44.7 ± 1.5	46.7 ± 1.5	*p* < 0.01	41 ± 1	45.3 ± 0.6	45.7 ± 2.1	*p* < 0.01

## Data Availability

All the available data are incorporated in the manuscript.
